The article "Deep Learning-Based Real-Time Discriminate Correlation Analysis for Breast Cancer Detection" was retracted in 2024. Reasons: signs of a paper mill; suspected computer-generated content; unreliable results or conclusions; concerns about the data.

# Deep Learning-Based Real-Time Discriminate Correlation Analysis for Breast Cancer Detection

**DOI:** 10.1155/2022/4609625

**Published:** 2022-06-28

**Authors:** Manisha Bhende, Anuradha Thakare, Bhasker Pant, Piyush Singhal, Swati Shinde, V. Saravanan

**Affiliations:** ^1^Marathwada Mitra Mandal's Institute of Technology, Pune, India; ^2^Pimpri Chinchwad College of Engineering, Pune, India; ^3^Department of Computer Science & Engineering, Graphic Era Deemed to Be University, Dehradun, Uttarakhand 248002, India; ^4^Department of Mechanical Engineering, GLA University, Mathura 281406, India; ^5^Department of Computer Engineering, Pimpri Chinchwad College of Engineering, Pune, India; ^6^Department of Computer Science, College of Engineering and Technology, Dambi Dollo University, Dambi Dollo, Oromia Region, Ethiopia

## Abstract

Breast cancer is the most common cancer in women, and the breast mass recognition model can effectively assist doctors in clinical diagnosis. However, the scarcity of medical image samples makes the recognition model prone to overfitting. A breast mass recognition model integrated with deep pathological information mining is proposed: constructing a sample selection strategy, screening high-quality samples across different mammography image datasets, and dealing with the scarcity of medical image samples from the perspective of data enhancement; mining the pathology contained in limited labeled models from shallow to deep information; and dealing with the shortage of medical image samples from the perspective of feature optimization. The multiview effective region gene optimization (MvERGS) algorithm is designed to refine the original image features, improve the feature discriminate and compress the feature dimension, better match the number of samples, and perform discriminate correlation analysis (DCA) on the advanced new features; in-depth cross-modal correlation between heterogeneous elements, that is, the deep pathological information, can be mined to describe the breast mass lesion area accurately. Based on deep pathological information and traditional classifiers, an efficient breast mass recognition model is trained to complete the classification of mammography images. Experiments show that the key technical indicators of the recognition model, including accuracy and AUC, are better than the mainstream baselines, and the overfitting problem caused by the scarcity of samples is alleviated.

## 1. Introduction

Authoritative reports show that breast cancer is the most common cancer in women and the second most deadly disease [1]. Therefore, breast lumps are a worrying breast abnormality, and about 90% of breast lumps are cancerous. Breast lumps are primarily hidden in breast tissue with unclear edges. Therefore, doctors must combine solid professional knowledge and rich diagnostic experience to complete accurate manual screening. However, doctors' diagnostic level is uneven, and manual screening is cumbersome and subjective, which can easily lead to a high rate of misdiagnosis or missed diagnosis. The computer-aided breast mass recognition model can effectively assist doctors in clinical diagnosis. However, as we all know, the vast majority of medical image processing applications are faced with the problem of sample scarcity. The main factors that cause this problem are as follows: (1) the cost of labeling medical images is too high, and it takes a lot of human resources and material resources to obtain a certain amount of high-quality samples; (2) due to the ethical clauses involved, a large number of medical image samples have personal privacy and cannot be obtained typically, which significantly limits the number of available samples; (3) due to the significant differences in the professional backgrounds involved, there is a particular “gap” between (medical) engineering (computer) cooperation, which in turn restricts the generation of high-quality samples. The scarcity of medical image samples can easily lead to fitting of the recognition model. In summary, how to deal with the shortage of medical image samples has become particularly important [2, 3]. In response to this problem, some scholars proposed to use the GAN (generative adversarial networks) model to generate new samples to expand the dataset, but the authenticity of the new selections was questioned; some scholars built a multitask learning framework (such as compound segmentation and recognition), that is, to deal with the scarcity of samples through information sharing between different tasks. Still, the design and training of multitask learning frameworks is complex [4, 5].

The article "Deep Learning-Based Real-Time Discriminate Correlation Analysis for Breast Cancer Detection" was retracted in 2024. Reasons: signs of a paper mill; suspected computer-generated content; unreliable results or conclusions; concerns about the data.

We are focusing on deep pathological information, which is a low-dimensional feature that has been mined numerous times, to fill the study gap. It has a lower dimension and is more discriminatory. It can better match the number of samples, lower the danger of model overfitting, and respond to medical imaging to a limited extent due to sample scarcity. It does not require the generation of new samples, and the model training is not complex, so the “cost-effectiveness” is higher than the other two approaches. As a result, we propose the “Breast Mass Recognition Model Integrated with Deep Pathological Information Mining” as a research topic. The deep pathological information in restricted labeled samples is mined from shallow to deep for training a high-quality and accurate model. Based on sample selection, the deep pathological information in limited labeled samples is mined from shallow through deep for training a high-quality and efficient breast mass recognition model. This paper contributes the following:

- Design a sample selection algorithm, select high-quality samples across different mammography image datasets, lay a data foundation for training a robust breast mass recognition model, and deal with the problem of sample scarcity from the perspective of data enhancement
- Design a multiview efficient range-based gene selection (MvERGS) algorithm, refine the original image features, and perform discriminate real time correlation analysis (DCA) to obtain the parts between the components [6]. The cross-modal correlation of the model is more discriminative. It has a lower dimension to match the number of samples, reduce the risk of model over fitting, and then deal with the problem of sample scarcity

The paper is organized into several sections where the first section states about the introduction of the problem followed by the second module, that is, the related work. The third section discusses about the proposed model framework, followed by the fourth section which states about the experiment and analysis. Finally, the end module discusses the conclusion of the work.

## 2. Related Work

### 2.1. Image Feature Learning

Image features are an essential prerequisite for breast mass recognition. Features such as scale-invariant feature transform (SIFT) and histogram of oriented gradients (HOG) have played an essential role in breast mass recognition [7, 8]. Literature extracted the image's interior and edge texture primitives and used linear discriminate analysis (LDA) to complete breast mass identification [9]. Literature optimized the critical features based on the mutual information model and used a support vector machine (SVM) to train the breast mass recognition model [9]. In addition, features such as complete local binary pattern (CLBP), grey-level cooccurrence matrix (GLCM), and other features have also been used for breast mass recognition [10, 11].

### 2.2. Feature Optimization

Because the feature dimension is high and contains noise, it is necessary to optimize the original image features to improve its discriminability and compress the feature dimension to better match the number of medical image samples. Feature optimization methods are divided into single-modal feature optimization and multimodal feature optimization as follows:

- Single-modal feature optimization literature extracted optical coefficients from optical tomography images as features and optimized features based on maximum correlation and minimum redundancy algorithms to complete rheumatoid arthritis detection [12]. Literature used a spatial grey difference feature extraction algorithm and correlation-based feature selection method to complete brain image classification [13]. Literature performed feature optimization based on particle swarm optimization (PSO) algorithm [14]. Literature improved the lion algorithm to select subsets of features such as texture, intensity histogram, and shape of breast images [15]. Literature combined LDA and local-preserving projection methods to optimize neuroimaging features [16]. The single-modal feature optimization method can refine the original features and improve the recognition accuracy
- Multimodal features preferably include positron emission tomography (PET), magnetic resonance imaging (MRI), computed tomography (CT), and other images so that they can surround them and expand multimodal feature optimization. Literature proposed a multimodal multitask learning framework to achieve multimodal feature fusion and complete diagnosis of Alzheimer's disease (AD) [17]. Literature performed latent feature learning for different modalities and mapped the features to the label space to complete AD diagnosis [18]. Literature used a sparse deep polynomial network (S-DPN) to complete multimodal data fusion to obtain new features with more robust discrimination [19]. Some scholars also use hypergraphs to complete high-order correlation analysis between multimodal data and generate high-quality features [20, 21]. The multimodal feature optimization method makes full use of the complementarity between features to improve the recognition accuracy

The article "Deep Learning-Based Real-Time Discriminate Correlation Analysis for Breast Cancer Detection" was retracted in 2024. Reasons: signs of a paper mill; suspected computer-generated content; unreliable results or conclusions; concerns about the data.

### 2.3. Breast Mass Recognition

In recent years, deep learning models have played an essential role in breast mass recognition. Mammograms are the most well-known tool for recognizing cancer in the breast at the initial stage. This cancer, which manifests itself mostly as mass, is hard to ascertain and diagnose because mass can be covered by normal breast tissue in breast density. Detection with the help of computers (CAD) is a method for avoiding mistakes in cancer screening of the breast, and its utility has been proven. Related work for breast mass recognition can be divided into four categories: fine-tuning model methods, ensemble deep learning methods, transfer learning methods, and multitask collaborative learning methods [22, 23]. The fine-tuning model method fine-tunes the pretrained convolutional neural network (CNN) to complete the recognition task. This method is simple and easy to use but is limited by the number of samples [24]. Literature connected the fully connected layer of the pretrained AlexNet model to the SVM to train the recognition model; the integrated deep learning method uses the complementarily between multiple models to improve recognition accuracy; this method requires a lot of computing resources [25]. Literature used DCNN (deep convolutional neural network) and deep belief network (DBN) to construct two prediction models, respectively and then integrated their results to realize breast mass recognition; the transfer learning method realizes recognition through a knowledge transfer task [26]. Literature used pretrained GoogLeNet, VGGNet, and ResNet models to extract image features, access the features to fully connected layers, pool them, and complete breast mass classification [27]. Literature first trained a patch-level recognition model, removed the fully connected layer, and added a new convolutional layer to train a recognition model for the entire angiographic image [28]. The multitask collaborative learning method refers to the diagnosis model including multiple related subtasks, such as lesion segmentation, tumor identification, and lesion localization, which complement each other, improve the recognition accuracy through collaborative learning, and reduce the dependence on the number of samples [29]. In summary, the lack of mammography images makes breast mass recognition more challenging [30]. The feature optimization algorithm can refine the original image features, better match the number of samples, and improve the model recognition performance. This paper proposes a “breast mass recognition model incorporating deep pathological information mining” to actively deal with the scarcity of medical image samples from multiple perspectives:

- Select high-quality samples across different mammography image datasets, laying the foundation for training a robust recognition model database
- Fully excavate the deep pathological information in the limited labeled samples to further alleviate the problem of model fitting: design the MvERGS algorithm to reduce noise interference and improve feature discrimination; in-depth analysis of the typical correlation between features, using cross-modal features to delineate the lesion area

To sum up, the model in this paper is called RMD, “R” stands for sample refinement, “M” stands for feature optimization algorithm MvERGS, and “D” stands for cross-modal analysis DCA. They are organically combined to improve breast mass recognition performance.

The article "Deep Learning-Based Real-Time Discriminate Correlation Analysis for Breast Cancer Detection" was retracted in 2024. Reasons: signs of a paper mill; suspected computer-generated content; unreliable results or conclusions; concerns about the data.

## 3. RMD Model Framework

The framework of the RMD model is shown in Figure 1, including sample selection, feature selection, cross-modal analysis, and breast mass recognition [31]. First, a sample selection strategy is designed to screen high-quality mammography image samples; second, SIFT (S), Gist (G), HOG (H), LBP (L), and DENSENET161 (D) are extracted from the perspectives of shape, texture, deep learning, etc., RESNET50(R) and VGG16(V) features. Third, consider feature diversity and complementarity, and lay the foundation for feature optimization and cross-modal analysis; design the feature optimization algorithm MvERGS to refine the original features and improve their discriminativeness, using $\tilde{\text{S}}$, $\tilde{\text{G}}$, $\tilde{\text{H}}$, $\tilde{\text{L}}$, $\tilde{\text{D}}$, $\tilde{\text{R}}$, and $\tilde{\text{V}}$, respectively; represent the new features after feature optimization; use the DCA method to analyze the cross-modal correlation between the new features; and generate cross-modal features, which are represented by “~SG,” “~SH,” “~SV,” “~GV,” etc. For example, “~SG” represents the cross-modal correlation between $\tilde{\text{S}}$ and $\tilde{\text{G}}$; the breast mass recognition model is trained based on cross-modal features and standard classifiers and outputs “0” and “1,” indicating negative and positive, respectively [32]. Furthermore, there may arise some drawbacks which emerge at reasonably high doses of radiation absorption such as tissue damage that include conjunctivitis, facial reddening, and baldness and are uncommon for several sorts of imaging methods.

### 3.1. Image Feature Extraction

Breast mass recognition necessitates the use of image feature extraction. Breast mass detection has relied heavily on features such the scale-invariant feature transform and the histogram of oriented gradient. The interior and edge texture primitives of the image were recovered, and linear discriminate analysis was employed to complete breast mass identification. Hence, this feature extraction plays a significant role in carcinoma detection where on the basis of ML techniques, essential features can be chosen based on the breast mass identification model. Image features should accurately describe the visual characteristics of breast mass and consider complementarily preparing for cross-modal analysis. For example, SIFT locates the variable shape of the mass; Gist depicts the texture characteristics of the mass from a global perspective; HOG captures the edge information of the mass to describe the appearance and shape of the mass; LBP depicts the texture changes of the mass from a local perspective. Deep learning features such as DENSENET161, RESNET50, and VGG16 are valuable supplements to standard components. The homologous network structure of the deep learning model was tried in the experiment, but the effect was slightly worse.

The article "Deep Learning-Based Real-Time Discriminate Correlation Analysis for Breast Cancer Detection" was retracted in 2024. Reasons: signs of a paper mill; suspected computer-generated content; unreliable results or conclusions; concerns about the data.

### 3.2. Sample Selection (R)

Breast mass recognition faces the problem of sample scarcity. Considering that randomly selecting samples to expand the dataset will introduce more noise information, which will affect the recognition performance of the model, try to choose samples with high confidence to expand the existing dataset, and reduce the impact of noise on recognition. Therefore, this paper designs a more targeted sample selection strategy, which spans different mammography image datasets, selects high-quality samples (confidence by a set of classifiers), and makes full use of the pathological knowledge contained in new instances [33, 34] to train a more effective and robust recognition model. To sum up, in the RMD model, the basic idea of the sample selection algorithm is to select a set of classifiers with the best performance and use a complex voting mechanism to choose samples from the source dataset; that is, the source dataset can be correctly classified by this set of classifiers. Finally, the pieces are selected and merged with the target dataset to train a new classification model. The idea is simple and easy to implement. It not only focuses on source samples with higher confidence but also makes full use of the complementarily of different classifiers in decision-making and finally lays a data foundation for training high-quality classification models.

### 3.3. Feature Optimization (M)

The selected samples in Section 3.2 are minimal and affected by individual differences. Fully mining the pathological information in tiny labeled pieces is a more effective method to deal with the problem of sample scarcity. This section scoops the pathological features of mammography images from the perspective of feature selection. The original image features have high dimensions and noise, which will affect the recognition accuracy and restrict the recognition efficiency. The MvERGS algorithm is designed to refine the original parts from two perspectives and improve their discriminativeness to deal with the model fitting problem caused by the scarcity of samples (the dimension will be significantly reduced after feature optimization to better match the number of pieces). At the same time, the algorithm has good expansibility. It can introduce more perspectives to more comprehensively and carefully describe the lesion area in the mammography image from a complementary perspective, improve the feature representation, and continuously enhance the discrimination of features, thereby improving the model recognition accuracy. Second, the algorithm is robust to a certain extent; it only processes the lowest-level feature components and does not depend on the visual content described by the features.

The article "Deep Learning-Based Real-Time Discriminate Correlation Analysis for Breast Cancer Detection" was retracted in 2024. Reasons: signs of a paper mill; suspected computer-generated content; unreliable results or conclusions; concerns about the data.

### 3.4. Cross-Modal Correlation Mining (D)

The MvERGS algorithm refines the original features, and the generated new features Fns contain shallow pathological information, which should further extract the deep pathological information in the labeled samples to better cope with the scarcity of samples. The texture, shape, color, edge, and other visual representations of similar breast masses point to the same or similar lesion area. The image features contain rich cross-modal correlation, which is of great significance for improving the recognition performance. Therefore, based on MvERGS feature optimization, we explore the cross-modal correlation between new features and continuously optimize the recognition accuracy.

## 4. Experiment and Analysis

### 4.1. Experimental Setup

#### 4.1.1. Dataset

Select public datasets CBIS-DDSM (https://wiki.cancerimagingarchive.net/display/ Public/CBIS -DDSM) and breast (http://medicalresearch.inescporto.pt/breastresearch/index.php/Get_INbreast_ Database) for experimental comparison, and their related information is shown in Table 1. For the breast dataset [35], images labeled 1 and 2 in BI-RADS are classified as negative samples, and images labeled 4, 5, and 6 are classified as positive samples. The PCA algorithm reduces SIFT and HOG to 500 and 300 dimensions. When extracting deep learning features, due to the large resolution, a significant cropping operation is performed on the image to make the input image 224 × 224. VGG16 selects the first fully connected layer with a feature dimension of 4096. Both DENSENET161 and RESNET50 select the last average pooling layer with feature dimensions of 2 208 and 2 048, respectively.

#### 4.1.2. Benchmark Algorithm

RMD models include RMD-KNN, RMD-LR, RMD-RF, RMD-DT, RMD-SVM, RMD-NB, RMD-Adaboost, RMD-GBDT, and RMD-XGBoost. There are five categories of comparison baselines, as follows:

- Mainstream feature optimization algorithms: GS-XGBoost, ERGS, Fisher Score, PSO, and HGSCCA [36]
- Recognition model based on MvERGS algorithm (M): M-KNN, M-LR, M-RF, M-DT, M-SVM, M-NB, M-Adaboost, M-GBDT, and M-XGBoost
- Identification models based on MvERGS algorithm (M) and cross-modal correlation mining (D): MD-KNN, MD-LR, MD-RF, MDDT, MD-SVM, MD-NB, MD-Adaboost, MD-GBDT, and MD-XGBoost
- Transfer learning class models: the models of DenseNet121, ResNet152, VGG16, and Literature [37]
- Recognition models based on regions of interest (ROI): the model of literature, the model of literature, the model of Zhu et al., the model of literature, and the model of literature [38]

The experimental results of (2) and (3) baselines can be regarded as performing ablation analysis on the RMD model. Since the category (5) baselines are based on ROI, indirect comparisons are made with these models. The performance of breast mass recognition was evaluated by indicators such as accuracy (Accuracy, Acc), AUC, sensitivity (Sensitivity, Sen), specificity (Specificity, Spe), and accuracy (Precision, Pre). The higher the accuracy and AUC, the better the recognition effect; the higher the sensitivity, the lower the false-negative rate, and the less missed diagnosis; the higher the specificity, the lower the false-positive rate, and the higher the diagnosis probability.

The article "Deep Learning-Based Real-Time Discriminate Correlation Analysis for Breast Cancer Detection" was retracted in 2024. Reasons: signs of a paper mill; suspected computer-generated content; unreliable results or conclusions; concerns about the data.

#### 4.1.3. Feature Robustness of MvERGS Algorithm

Extract the single category features “S,” “G,” “H,” “L,” “D,” “R,” and “V,” and complete the identification task based on the traditional classifier. Take the best results of each feature on the classifier for display and experimental results, as shown in Table 2. In the CBIS-DDSM dataset, the S feature performs well, with a false-positive rate of only 1.39%. The S feature can reduce the noise caused by changes in morphology and viewing angle and help the model lock the breast mass's shape accurately. Second, G features capture abnormally textured breast masses from a global perspective. In TP “TN,” the model is prone to overfitting. In the breast dataset, D features and V features outperform. The number of positive predictive samples is much smaller than the number of negative predictive samples (TP+FP “TN”+FN), or the predictive probability of positive samples is 0 (PrePos=0), and the recognition model has serious overfitting, and the scarcity of samples is the cause of this and is the most important factor in the results [39]. Therefore, using high-dimensional original features for breast mass recognition, the overall recognition performance is not good due to overfitting. This requires fully excavating the low-dimensional and deep pathological information contained in the original image, features, more accurately depicting the lesion area of the mammography image, and matching the number of samples to reduce the risk of model overfitting [40]. Therefore, the RMD model proposed in this paper can mine valuable pathological information from shallow to deep, thereby improving the recognition performance and actively dealing with the problem of sample scarcity. Based on the MvERGS algorithm, feature optimization is performed on the original image features such as “S,” “G,” “H,” “L,” “D,” “R,” and “V” in Table 2, and new features “$\tilde{\text{S}}$,” “$\tilde{\text{G}}$,” and “$\tilde{\text{H}}$” are generated [41]. “$\tilde{\text{L}}$,” “$\tilde{\text{D}}$,” “$\tilde{\text{R}}$,” and “$\tilde{\text{V}}$” compare fairly and fully verify the importance of the feature optimization algorithm, the common classifier is still selected to complete the breast mass recognition, and the optimal result of each feature is displayed on the classifier. This demonstrates the MvERGS algorithm's scalability, implying that additional views can be absorbed into it to boost its efficiency, even more. Second, it only works with certain types of data. The bottom has components and is independent of the top, including the visual material to a high degree. This demonstrates the system's sturdiness and MvERGS algorithm, demonstrating that it is capable of high performance computing any feature in any field of investigation. As a consequence, the MvERGS numerous subsequent scientific disciplines can benefit from the algorithm that necessitates elaborate features. The experimental results are shown in Table 3, and “↑” indicates an improvement compared to the results in Table 2. Avg1 represents the mean value of all indicators of the original image features on the CBIS-DDSM dataset (calculated based on Table 2), Avg2 represents the mean value of all indicators of the new features on the CBIS-DDSM dataset, and Avg3 represents the original image features on the breast dataset [42]. The mean of all indicators (calculated based on Table 2) and Avg4 represents the mean of all indicators of new features on the breast dataset (calculated based on Table 3). Calculating these quantities can better judge the merits of the MvERGS algorithm. Figures 2 and 3 show the accuracy and productivity over robustness feature.  Figure 4 shows the confusion element over robustness feature.

The article "Deep Learning-Based Real-Time Discriminate Correlation Analysis for Breast Cancer Detection" was retracted in 2024. Reasons: signs of a paper mill; suspected computer-generated content; unreliable results or conclusions; concerns about the data.

In the CBIS-DDSM dataset, (1) after feature optimization, the recognition performance of other new features has been improved except for the “$\tilde{\text{G}}$” feature, among which the “$\tilde{\text{L}}$” feature acc has the most significant improvement (10.53 percentage points), and its AUC has also improved effective (13.67 percentage points). The MvERGS algorithm refines the original features and enhances their discriminativeness. (2) The S feature is the best before the MvERGS algorithm is implemented, and the “$\tilde{\text{S}}$” feature is still the best after the feature is optimized, the false-positive rate is reduced to 0.93%, 2.47 percentage points increase the AUC value, and the practicability of the model is continuously improved. The MvERGS algorithm is effective, and it preserves the core components of the original features to the greatest extent. This shows that fully mining the deep pathological information in the limited labeled samples can improve the model recognition performance. (3) From the perspective of mean value, all indicators have been improved after feature optimization. AUC and ACC have improved significantly, reaching 3.01 percentage points and 2.51 percentage points, respectively. The overall recognition performance of the model is better, indicating that the MvERGS algorithm is robust. More importantly, TP is gradually increasing, FN is slowly decreasing, and the overfitting tendency of the breast mass recognition model has been corrected to a certain extent; that is, new features with more compact dimensions can better match the number of training samples to cope with the scarcity of pieces. In summary, the MvERGS algorithm is effective on the CBIS-DDSM dataset, which verifies the integrity of the valuable information in the FN feature from another aspect. Figures 5 and 6 show the accuracy and productivity over MvERGS algorithm. The confusion element over MvERGS algorithm is shown in Figure 7.

The article "Deep Learning-Based Real-Time Discriminate Correlation Analysis for Breast Cancer Detection" was retracted in 2024. Reasons: signs of a paper mill; suspected computer-generated content; unreliable results or conclusions; concerns about the data.

In the breast dataset, (1) after feature optimization, all feature recognition performances have been improved, among which the “$\tilde{\text{R}}$” feature acc has improved significantly (4.31 percentage points), and its AUC value has been dramatically improved (22.49 percentage points). In terms of AUC improvement, the breast dataset performs better. Since the mammography images of the breast are more precise, the MvERGS algorithm can better refine the original features, thus laying an essential foundation for training an excellent recognition model. (2) After feature optimization, “n” “$\tilde{\text{S}}$” has the best overall performance, and 6.37 percentage points increase its AUC value. This shows that the noise information is indeed less after feature optimization, and the new features can more accurately describe the visual characteristics of the image. (3) The overfitting of the model is alleviated to a certain extent. The number of samples in the breast dataset is small and unbalanced, and many original features are overfitted. After implementing the feature optimization based on the MvERGS algorithm, the discriminative of new features is enhanced, the TP, FN, and other indicators are significantly improved, the number of misclassified samples is continuously reduced, and the tendency of overfitting is alleviated. (4) Measured from the mean point of view, most of the indicators have been improved after feature optimization (compared to the CBIS-DDSM dataset, three indicators have not been improved, and the breast dataset is more challenging, which also shows that data scarcity affects the identification of impact), such as PrePos, Sen, and AUC, and the improvement of the PrePos indicator is also a vital sign that the overfitting problem is alleviated. To sum up, the MvERGS algorithm is also effective on the breast dataset, which verifies the integrity of the valuable information in the FN features from another aspect. To sum up, after MvERGS feature optimization, the recognition performance on both datasets has been improved. The overfitting has been alleviated to a certain extent. Of course, the indicators such as sensitivity and accuracy on the two datasets are still low. It is necessary to continue performing cross-modal correlation mining to improve these indicators.

The article "Deep Learning-Based Real-Time Discriminate Correlation Analysis for Breast Cancer Detection" was retracted in 2024. Reasons: signs of a paper mill; suspected computer-generated content; unreliable results or conclusions; concerns about the data.

#### 4.1.4. Essential Indicators of the RMD Model

In clinical diagnosis, specificity and sensitivity are also essential. The higher the specificity, the lower the false-positive rate, and the higher the probability of diagnosis; the higher the sensitivity, the lower the false-negative rate, the less missed diagnosis, and the actual patients can be treated in time. Specificity and sensitivity assess model utility from different perspectives. Draw the change graph of the specific mean and sensitivity mean of the RMD model as shown in Figure 4. The orange column represents the increase, the green column represents the decrease, and the blue column represents the mean. If the orange column is included, the blue column, the sum of the height of the orange bar, is the mean value of the corresponding indicator. The blue column represents the mean value of the corresponding index after introducing the sample selection strategy.

Selecting the mean can discover the real trend from a statistical point of view. “breast➝DDSM” indicates the direction of sample selection, that is, selecting samples from the breast dataset to supplement the DDSM dataset. “DDSM ➝breast” means just the opposite. On the CBIS-DDSM dataset, cross-modal features containing “$\tilde{\text{S}}$” have higher specificity. This means that the number of misdiagnosed patients is decreasing, which can ease the psychological burden of partients. After implementing the sample selection strategy, the specificity of 10 sets of cross-modal features was improved, of which “~SH” and “~LD” improved significantly. This shows that the features such as “$\tilde{\text{D}}$” and “$\tilde{\text{L}}$” of the samples selected from the breast can better explain the samples in CBIS-DDSM, thereby improving the model specificity. On the breast dataset, the specificity improvement was not significant, and after implementing the sample selection strategy, the specificity of the five cross-modal features was improved. After all, there are specific differences between the individuals corresponding to the two types of samples, CBIS-DDSM and breast, and the image resolution and clarity are also different. On the CBIS-DDSM dataset, cross-modal features containing “$\tilde{\text{S}}$” have higher sensitivity. After implementing the sample selection strategy, the sensitivity of 6 groups of cross-modal features is improved, of which “a ~GD” and “~HD” are significantly improved, and the deep learning feature “$\tilde{\text{D}}$” plays an important role. This shows that the features such as “$\tilde{\text{D}}$” and “$\tilde{\text{L}}$” of the selected samples from the breast are beneficial supplements to the CBIS-DDSM dataset, which is consistent with the conclusion in Figure 4. The “$\tilde{\text{D}}$” feature has strong robustness. On the breast dataset, most cross-modal features show better sensitivity. The cross-modal features containing “$\tilde{\text{S}}$” and “$\tilde{\text{R}}$” perform the best. After implementing the sample selection strategy, the sensitivity of the 13 groups of cross-modal features was improved. The sensitivity of the breast dataset is significantly enhanced. The pathological knowledge extracted from CBISDDSM can better describe the visual characteristics of negative samples, the false-negative rate is reduced, and the sensitivity is improved, which helps reduce the phenomenon of missed diagnosis and reduce the actual cost.

The article "Deep Learning-Based Real-Time Discriminate Correlation Analysis for Breast Cancer Detection" was retracted in 2024. Reasons: signs of a paper mill; suspected computer-generated content; unreliable results or conclusions; concerns about the data.

In summary, for a dataset with more balanced samples, the RMD model can obtain better specificity, which helps to reduce the false-positive rate of diagnosis and improve the diagnosis rate. On the other hand, for datasets with relatively low samples, the RMD model can obtain better sensitivity, which helps to reduce the phenomenon of missed diagnosis and reduce the cost to patients. Clearly, after introducing the sample selection strategy, the specificity and sensitivity of the recognition model show positive changes, which enhance the practicability of the model to a certain extent.

## 5. Conclusion

In this work, we propose a breast mass recognition model RMD that is coupled with deep pathological information mining in this paper. Because the breast mass recognition model would aid doctors in clinical diagnosis, but there are not enough samples, the recognition accuracy will be limited, limiting the model's applicability. As a result, from the perspectives of sample selection, feature selection, and cross-modal correlation mining, this work actively reacts to the challenge of sample scarcity. Experiments indicate that the RMD model optimizes the recognition accuracy on two general mammography picture datasets, and that each component of the model (R, M, D) is useful. The most notable feature of the RMD model is to perform multistage, layer-by-layer feature selection to gain new features with stronger discriminative and lower dimensions. Of course, the RMD model is not end-to-end. As a result of this model, a web-based breast cancer diagnosis platform was created and internal testing was completed. Feature extraction, sample selection, feature optimization, and cross-modal correlation mining are all included in the platform. The technology is expected to speed up the model's actual landing, allowing doctors to make better clinical diagnoses. The nonlocal block model will be offered in the future to complete the localization of breast mass based on mass breast identification; additionally, the RMD model is likely to be used to detect new coronary pneumonia.

The article "Deep Learning-Based Real-Time Discriminate Correlation Analysis for Breast Cancer Detection" was retracted in 2024. Reasons: signs of a paper mill; suspected computer-generated content; unreliable results or conclusions; concerns about the data.

## Figures and Tables

**Figure 1:** Proposed model.

**Figure 2:** Accuracy over robustness feature.

**Figure 3:** Productivity over robustness feature.

**Figure 4:** Confusion element over robustness feature.

**Figure 5:** Accuracy over MvERGS algorithm.

**Figure 6:** Predicatively over MvERGS algorithm.

**Figure 7:** Confusion element over MvERGS algorithm.

**Table 1:** Detail description of dataset.

Dataset	After preprocessing size/pixel	Negative samples/frame	Positive samples/frame	Train-test ratio
CBIS-DDSM	1152 × 896	1434	1347	70%-30%
INbreast	2500 × 3300	287	100	

**Table 2:** Performance evaluation over original image feature.

	Feature	Accuracy	Predicted positive	Predicted negative	Sensitivity	Specificity	AUC
CBIS-DDSM	S	82.56	74.56	64.62	60.28	89.56	95.52
	G	75.23	72.54	61.45	58.26	84.26	85.63
	H	70.26	68.26	60.84	54.56	82.51	74.26
	L	68.36	62.48	57.36	52.24	80.59	64.56
	D	65.26	59.23	55.62	50.68	80.24	56.34
	R	64.25	58.42	52.6	49.52	78.56	55.28
	V	59.56	52.56	50.85	48.56	76.85	50.28

INbreast	S	80.26	78.56	68.65	69.26	94.65	92.58
	G	74.26	74.52	65.25	68.45	92.68	90.86
	H	72.28	72.58	64.86	67.28	90.84	76.25
	L	65.78	68.48	59.62	61.24	88.63	69.25
	D	60.86	64.26	54.26	58.67	86.54	58.26
	R	59.56	59.85	52.26	56.95	84.68	55.28
	V	55.68	54.87	51.25	55.28	82.98	51.45

**Table 3:** Performance evaluation over MvERGS algorithm.

	Feature	Accuracy	Predicted positive	Predicted negative	Sensitivity	Specificity	AUC
CBIS-DDSM	S	80.91	73.81	62.04	54.85	84.19	94.56
	G	73.73	71.81	58.99	53.02	79.20	84.77
	H	68.85	67.58	58.41	49.65	77.56	73.52
	L	66.99	61.86	55.07	47.54	75.75	63.91
	D	63.95	58.64	53.40	46.12	75.43	55.78
	R	62.97	57.84	50.50	45.06	73.85	54.73
	V	58.37	52.03	48.82	44.19	72.24	49.78

INbreast	S	78.65	77.77	65.90	63.03	88.97	91.65
	G	72.77	73.77	62.64	62.29	87.12	89.95
	H	70.83	71.85	62.27	61.22	85.39	75.49
	L	64.46	67.80	57.24	55.73	83.31	68.56
	D	59.64	63.62	52.09	53.39	81.35	57.68
	R	58.37	59.25	50.17	51.82	79.60	54.73
	V	54.57	54.32	49.20	50.30	78.00	50.94

The article "Deep Learning-Based Real-Time Discriminate Correlation Analysis for Breast Cancer Detection" was retracted in 2024. Reasons: signs of a paper mill; suspected computer-generated content; unreliable results or conclusions; concerns about the data.

## Data Availability

The data shall be made available on request.

## References

[1] Orel V. E., Rykhalskyi O., Syvak L. (2020). Computer-assisted inductive moderate hyperthermia planning for breast cancer patients.

[2] Burriel V., Pastor O., Pena-Chilet M., Martinez M. T., Ribas G. (2016). Conceptual schema of miRNA’s expression: using efficient information systems practices to manage and analyse data about miRNA expression studies in breast cancer.

[3] Burriel V., Pastor O., Peña-Chilet M., Martínez M. T., Ribas G. Conceptual schema of miRNA's expression: using efficient information systems practices to manage and analyse data about miRNA expression studies in breast cancer.

[4] Bilgic B. Comparison of breast cancer and skin cancer diagnoses using deep learning method.

[5] Park K., Chen W., Chekmareva M. A., Foran D. J., Desai J. P. (2018). Electromechanical coupling factor of breast tissue as a biomarker for breast cancer. *IEEE Transactions on Biomedical Engineering*.

[6] Easson A., Pandya A., Pasternak J., Mohammed N., Douplik A. (2020). Improving the patient cancer experience: multispectral (white light/autofluorescence/Raman) needle endoscopy for cancer diagnostics in breast and thyroid.

[7] Mahrooghy M., Ashraf A. B., Daye D. (2015). Pharmacokinetic tumor heterogeneity as a prognostic biomarker for classifying breast cancer recurrence risk. *IEEE Transactions on Biomedical Engineering*.

[8] Keatmanee C., Makhanov S. S., Kotani K., Lohitvisate W., Thongvigitmanee S. S. Automatic initialization of active contour model in breast cancer detection utilizing conventional ultrasound and Color Doppler.

[9] Li Q., Xiao X., Wang L. (2015). Direct extraction of tumor response based on ensemble empirical mode decomposition for image reconstruction of early breast cancer detection by UWB. *IEEE Transactions on Biomedical Circuits and Systems*.

[10] Tripathi A., Misra K. Stilbene analogues as inhibitors of breast cancer stem cells through P-glycoprotein efflux; A 3D quantitative structure-activity relationship study (inhibitory activity of stilbenes analogues on breast cancer stem cells).

[11] Amkrane Y., El Adoui M., Benjelloun M. Towards breast cancer response prediction using artificial intelligence and radiomics.

[12] Aibe N., Karasawa K., Aoki M. (2019). Results of a nationwide survey on Japanese clinical practice in breast-conserving radiotherapy for breast cancer. *Journal of Radiation Research*.

[13] Li M. Research on the detection method of breast cancer deep convolutional neural network based on computer aid.

[14] Hagness S. C., Taflove A., Bridges J. E. (1998). Two-dimensional FDTD analysis of a pulsed microwave confocal system for breast cancer detection: fixed-focus and antenna array sensors. *IEEE Transactions on Biomedical Engineering*.

The article "Deep Learning-Based Real-Time Discriminate Correlation Analysis for Breast Cancer Detection" was retracted in 2024. Reasons: signs of a paper mill; suspected computer-generated content; unreliable results or conclusions; concerns about the data.

[15] Reis S., Gazinska P., Hipwell J. H. (2017). Automated classification of breast cancer stroma maturity from histological images. *IEEE Transactions on Biomedical Engineering*.

[16] Botterill T., Lotz T., Kashif A., Chase J. G. (2014). Reconstructing 3-D skin surface motion for the DIET breast cancer screening system. *IEEE Transactions on Medical Imaging*.

[17] Kao T.-J. (2008). Regional Admittivity spectra with tomosynthesis images for breast cancer detection: preliminary patient study. *Institute of Electrical and Electronics Engineers (IEEE)*.

[18] Portieri A., Grootendorst M., Fitzgerald T. Intra-operative terahertz probe for detection of breast cancer.

[19] Sayed S., Ahmed S., Poonia R. Holo entropy enabled decision tree classifier for breast cancer diagnosis using Wisconsin (prognostic) data set.

[20] Liu T., Zhou L., Rong W. Real-time PCR and immunohistochemistry detecting the expression of PETA-3 in breast cancer and the clinical significance.

[21] Umesh D. R., Ramachandra B. Association rule mining based predicting breast cancer recurrence on SEER breast cancer data.

[22] Gamagami P., Silverstein M. J., Waisman J. R. Infra-red imaging in breast cancer.

[23] Khasana U., Sigit R., Yuniarti H. Segmentation of Breast Using Ultrasound Image for Detection Breast Cancer.

[24] Bowman T., El-Shenawee M., Bailey K. Terahertz time-domain pulsed spectroscopy of human breast cancer tissues.

[25] Ara S., Das A., Dey A. (2021). Malignant and benign breast cancer classification using machine learning algorithms.

[26] Yifan D., Jialin L., Boxi F. Forecast model of breast cancer diagnosis based on RF-AdaBoost.

[27] Song H., Sasada S., Masumoto N. (2019). Detectability of breast tumors in excised breast tissues of Total mastectomy by IR-UWB-radar-based breast cancer detector. *IEEE Transactions on Biomedical Engineering*.

[28] Khuriwal N., Mishra N. Breast cancer diagnosis using adaptive voting ensemble machine learning algorithm.

[29] Atif M., AlSalhi M. S., Devanesan S., Masilamani V., Farhat K., Rabah D. Spectral characterization of breast cancer.

[30] Rosenthal D. T., Iyer H., Escudero S. From in vitro to in silico and back again: Using biological and mathematical synergy to decipher breast cancer cell motility.

[31] Yao Q., Shabaz M., Lohani T. K., Wasim Bhatt M., Panesar G. S., Singh R. K. (2021). 3D modelling and visualization for vision-based vibration signal processing and measurement. *Journal of Intelligent Systems*.

[32] Dhondalay G. K., Tong D. L., Ball G. R. Estrogen receptor status prediction for breast cancer using artificial neural network.

The article "Deep Learning-Based Real-Time Discriminate Correlation Analysis for Breast Cancer Detection" was retracted in 2024. Reasons: signs of a paper mill; suspected computer-generated content; unreliable results or conclusions; concerns about the data.

[33] Vesnin S., Goryanin I. (2017). Modern microwave thermometry for breast cancer. *Journal of Molecular Imaging & Dynamics*.

[34] Byrne D., O’Halloran M., Jones E., Glavin M. A comparison of data-independent microwave beamforming algorithms for the early detection of breast cancer.

[35] Nagpure R., Chandak S., Pathak N. Breast cancer detection using neural network mammogram.

[36] Almarzouki H. Z., Alsulami H., Rizwan A., Basingab M. S., Bukhari H., Shabaz M. (2021). An internet of medical things-based model for real-time monitoring and averting stroke sensors. *Journal of Healthcare Engineering*.

[37] Gupta A., Kapoor L., Wattal M. (2011). C2c (cloud-to-cloud): An ecosystem of cloud service providers for dynamic resource provisioning. *International Conference on Advances in Computing and Communications*.

[38] Chaudhury S., Shelke N., Sau K., Prasanalakshmi B., Shabaz M. (2021). A novel approach to classifying breast cancer histopathology biopsy images using bilateral knowledge distillation and label smoothing regularization. *Computational and Mathematical Methods in Medicine*.

[39] Robinson D. S., Manns F., Parel J. M. A clinical approach to the development of interstitial therapy of primary breast cancer.

[40] Gupta A. Performance insight 360: A cloud-based quality management framework for educational institutions in India.

[41] Thakur T., Batra I., Luthra M. (2021). Gene expression-assisted cancer prediction techniques. *Journal of Healthcare Engineering*.

[42] Fu B., Liu P., Lin J., Deng L., Hu K., Zheng H. (2019). Predicting invasive disease-free survival for early stage breast cancer patients using follow-up clinical data. *IEEE Transactions on Biomedical Engineering*.

